The article "Does Green Financing Develop a Cleaner Environment for Environmental Sustainability: Empirical Insights From Association of Southeast Asian Nations Economies" was retracted in 2025. Reasons: unreliable results or conclusions; a conflict of interest; concerns about the peer review; concerns about the citations.

# Does Green Financing Develop a Cleaner Environment for Environmental Sustainability: Empirical Insights From Association of Southeast Asian Nations Economies

**DOI:** 10.3389/fpsyg.2022.904768

**Published:** 2022-06-16

**Authors:** Weiwei Fu, Muhammad Irfan

**Affiliations:** ^1^School of Finance, Southwestern University of Finance and Economics, Chengdu, China; ^2^School of Management and Economics, Beijing Institute of Technology, Beijing, China; ^3^Centre for Energy and Environmental Policy Research, Beijing Institute of Technology, Beijing, China; ^4^Faculty of Management Sciences, Department of Business Administration, ILMA University, Karachi, Pakistan

**Keywords:** cleaner environment, green financing, climate change, environmental sustainability, ASEAN economies

## Abstract

One of the most frequently used terms in climate change discussions is environmental sustainability. With economic growth and foreign direct investment as moderator factors, this study investigates the influence of green finance and financial development on environmental sustainability and growth in ASEAN economies from 2012 to 2019. ADF and Phillip-Peron (PP) unit root tests, fully modified least square (FMOLS), were employed for long-run empirical estimates. A substantial body of evidence supports the study’s findings using VECM technology. Green financing was negatively associated with CO2 emissions. However, environmental sustainability in ASEAN is favorably associated with green financing. It is also worth noting that green financing promotes environmental sustainability at the expenditure of economic growth. Financial development, foreign direct investment, R&D investment, and green technology foster economic expansion at the price of environmental sustainability. There are still many fences to green finance that need to be addressed, including pricing CO2 emissions and reforming inefficient nonrenewable fossil fuel subsidies. Local governments play a vital role in eliminating these barriers and addressing disincentives. It is recommended that policymakers push the financial sector to adopt a green finance strategy to further the goals of long-term sustainable development. Industry must integrate multiple objectives, such as inclusive growth and environmental protection and productivity, through an even broader range of legislative frameworks ideal for decoupling growth from social and ecological unsustainability, at the heart of the green manufacturing process.

## Introduction

Indonesia, Malaysia, Singapore, and Thailand molded the Association of Southeast Asian Nations (ASEAN) in July 1967 to endorse economic development, social improvement, and cultural development. It began in 1984 with Brunei, followed by Vietnam in 1995, Laos and Myanmar in 1997, and other countries. One million square miles and more than 600 million people populate the ASEAN region (4.5 million km^2^). For example, ASEAN’s most important initiatives include joint research and technology cooperation programs among member countries under cooperative peace and shared prosperity (Huang X. et al., 2022). This regional organization’s most significant efforts are centered on the expansion of commerce between ASEAN countries and other countries and programs for joint scientific research and technology cooperation among the member governments. Some have challenged growing regional integration as threatening international institutions and isolating governments outside the region (Feng H. et al., 2022; Rao et al., 2022; Xiang et al., 2022a). They fear this will happen. After the Asian financial crisis of 1997–1998, it is suggested that liquidity come from outside the area. As a result of this, the Chiang Mai Agreement has spurred the development of a truly multilateral organization for bilateral swap agreements and the creation of an Asian currency.

For centuries, the financial industry has served as a tremendous force for human advancement (Nureen et al., 2022; Xie et al., 2022). Savings from all across the world must be used wisely, and here is where the global financial system comes in handy (Irfan et al., 2020a). People’s quality of life can be improved with the proper use of investment (Iqbal et al., 2020; Irfan et al., 2020b; Iqbal W. et al., 2021; Xiang et al., 2022b). Many people have put their funds in environmentally hazardous ventures and real-estate bubbles as a result of the collapse of the banking system (Rehman et al., 2020). As a result of the financial sector’s previous disregard for the ecosystem, environmental problems such as territory loss and resource lessening (Ahmad M. et al., 2021; Fang et al., 2022; Irfan et al., 2022a), environment change (Dagar et al., 2022; Islam et al., 2022), and effluence have emerged or worsened (Irfan et al., 2022b).

Although the importance of finance in the anthropogenic (i.e., human influence on the ecosystem), slight has been done to merge environmental problems into finance (Tawiah et al., 2021). In recent years, investments in sustainable growth have received more attention from the financial sector (Wu et al., 2021). Green financial products, according to Habiba and Xinbang (2022), can aid in the creation of a greener world. The terms green finance and sustainable finance are interchangeable, as are climate finance. Investments that improve the environment are referred to as green finance (Yang et al., 2021; Chishti and Sinha, 2022). On the other hand, climate finance is financing that attempts to sustenance climate change mitigation and adaptation efforts (Abbas et al., 2020; Chien F. S. et al., 2021; Yu et al., 2022). Financing tools for sustainable development are what bind all of these terms together. Investing in renewable and clean energy projects is essential for reducing carbon emissions and their harmful effects on human health and the environment (Irfan and Ahmad, 2021, 2022). It incorporates environmental considerations into financial decision-making. These environmental and sustainability considerations will be enhanced through the use of green finance to fund climate-neutral as well as resource-efficient technologies (Bhardwaj et al., 2022).

In recent years, green finance has also gained much attention as an emergent paradigm of finance development (Mikhno et al., 2021; Chen et al., 2022). Green finance and finance have become problematic terms in this context. According to Abbasi et al. (2022), green finance is a new financial pattern that combines environmental conservation with economic profit. Eco-friendly finance is an essential component of the transition to sustainability, and its development aims to reinforce particular financial features to enhance environmental quality (Wei et al., 2022). As of this writing, academics have centered on the fundamentals of green finance, such as how to integrate environmental protection into finance (Tang et al., 2022) and how to build green finance operating mechanisms within environmental protection systems (Sun et al., 2021), and the role of government in green finance implementation (Franco et al., 2021). Empirical investigations on the connection between green finance and the environment also play a role in this topic. A recent study by Weihong et al. (2021) indicated that lessening carbon emissions by using green financing policies had a favorable impact. However, the effects were short-lived and lacked continuity. Green economic growth is facilitated by the public from green finance, as Chien F. et al. (2021) have demonstrated. When applying the spatial econometric model, Nasir et al. (2022) discovered green finance’s environmental spillover effects. Green bonds, green loans, greenhouse mortgages for commercial buildings, ecological home equity programs, go green auto loans, Small and medium-size enterprises expedited loans, and climate credit cards have been developed by financial intermediaries and markets. Australians also started a long-term financial mechanism called the Environmental Deposit Initiative, which aims to assist climate change and sustainable development by providing medium- to long-term funding for environmentally friendly company ventures.

Few studies look at regional heterogeneity and factors that drive green finance and environmental sustainability to evolve in concert. This is obvious from examining the previous studies on green finance and environmental sustainability. According to a literature assessment, green finance has thus far been measured using a pretty straightforward method. Most academics use one or two indicators, which lack a broad perspective. The originality of this study is based on the fact that: As part of the global fight for efficient resource allocation and sustainable development, this article attempts to highlight the importance of developing a green financial system. As a result, economic growth can protect and improve the environment (Saha et al., 2022). There are still considerable hurdles to overcome in developing a green financial market, even though it improves resource allocation efficiency and accelerates the transition to a more sustainable growth model.

Green financial solutions aren’t all the same, and there aren’t as many options as there used to be. Green businesses are hindered because a single product can be defined in various ways (Zhang et al., 2021). ASEAN’s growth has been primarily driven by the green credit and green bond markets. Although new green financial products can draw public money third-party authorization bodies lack a clear definition of the standards for evaluating green initiatives, simply leading to the phenomenon that green projects are expelled by non-low-carbon projects (Mngumi et al., 2022).

While there are positive externalities and good environmental advantages to green projects, An et al. (2021), When compared to more traditional projects, green ones suffer from a lack of necessary skills and a high initial cost (Feng S. et al., 2022). Enterprises’ passion for green creation will decline if there is less assistance from the green project intermediary, information services, and other specialized organizations. There is a demand for innovative financial and ecological economics expertise in developing green financing. A scarcity of qualified individuals hampers sustainable growth in green finance.

The aim of the study is to investigate the impact of green finance on environmental sustainability. Heterogeneous interests characterize green financial engagement (Wang et al., 2021). Policy and regulations developed by the ASEAN promote green finance. As a result, ASEAN incentives and involvements do not substantially address the issue of the green driving force in firms (Ning et al., 2021). So it will be tough to execute the policy system (Mastini et al., 2021). The only option is to go for the highest possible profit margin for businesses. A dynamic green financial market relies heavily on financial institutions. Market activity is minimal, and revenues aren’t very large because innovative financial products are easy to understand (Li et al., 2022). Encouraging the flow of social capital into green financial markets is a difficult task. Consumers purchase green items according to utility maximization (Huang H. et al., 2022). Green financial markets can’t grow if consumers aren’t encouraged to participate in environmental conservation through the correct use of subsidies.

The rest of the article is organized as follows: Section “Literature Review” offers a brief overview of relevant literature and outlines the research’s primary findings. Introducing the green finance operating mechanism, defining parameter notations, making corresponding assumptions and building a basic evolutionary of the interactions between a clean environment, foreign direct investment (FDI), financial institutions and environmental sustainability are all covered in Section “Methodology.” Varied incentives have different effects on VECM and FMOLS outcomes in Section “Results and Discussion.” Simulates and analyses the long-term viability and strategy of green financing and its impact on participating entities. Section “Conclusion and Policy Implications” concludes the discussion.

## Literature Review

### The Connotation of Green Finance

Research on green finance in international academics often goes through four stages: the emergence of green finance, sturdy development, surging growth and speedy growth. From 1998 to 2002, the notion of green finance was developed. According to Ning et al. (2022), Green finance is a vital link between the financial and environmental industries and critical financial innovation in the quest for environmental conservation. The green finance theory underwent a steady evolution between 2000 and 2005. For (Jinru et al., 2021), environmental protection was the starting point for developing the theoretical foundations of finance, which included the financial services industry as a distinct service sector. Green finance theory went through a rough patch between 2006 and 2011. Financial organizations are developing green financial services in underdeveloped nations and emerging international nations. Anh Tu et al. (2021) performed surveys and in-depth explorations and assessments on regional environmental investment. The notion of green finance was rapidly evolving in 2012. Rights price marketplaces, individual investors’ knowledge, and financial institutions’ sustainability in the development of the green company were all explored. These findings demonstrate that foreign researchers’ knowledge of green finance has evolved from phenomenon to essence, from simple to complex. This growth has occurred in tandem with the growing worldwide awareness of environmental challenges. Ecological sustainability is the goal of a green economy, defined by Jinru et al. (2021) as the coordinated development of those above three.

Compared to academic circles in other nations, domestic research into green finance theory began later in the United States. There are primarily three representative viewpoints on what it means to do green finance: According to Zhang et al. (2021), green finance is a special financial policy that prioritizes the provision of financial services to environmentally friendly and clean businesses. According to Nawaz et al. (2021), green finance needs the financial industry to safeguard the environment. Sun et al. (2022) defined green finance as a financial instrument novelty designed for environmental protection. On the other hand, the third viewpoint is more comprehensive and has gained widespread acceptance in the academic world here in the United States. There are numerous studies out there looking at green finance from this standpoint. Zhang and Vigne (2021) studied green finance’s meaning, dimension, and structure. With the help of data from six central Chinese provinces, Zhang and Vigne (2021) employed a fixed-effect model to examine the impact of green funding on provincial economic development and proposed appropriate remedies.

### The Environmentalization of the Association of Southeast Asian Nations Economy

Humans have a strong desire to sustain stability between the economy and the environment, leading to the environmentalization of the economy. It is a decision-making science investigating economic progress and inter-regional links from a macro level. Kenneth Boulding, an American economist, was the first to propose it in 1966. He argues that environmental economics is a subject that analyses the interaction between environmental systems and economic structures and encompasses modern-day environmental economics and regulations touched by green financing. The economic growth model will lead to resource reduction, ecological deterioration, and finally, economic collapse if it is based solely on growth. As Sun et al. (2022) showed, the study region’s renewable energy sector’s financial development has been a substantial positive element of the renewable energy sector in the study area. Using the objective rules of ecosystems and ecological processes, Jin et al. (2021) contend that humans must control and regularize the natural environments in which they live. Ning et al. (2022) said that the mechanical study technique shows that the economic-centric development model will ultimately lead to the nations’ economic crisis if the ecological rules are violated, and the ecosystem is damaged. The ecological economy can only be realized if methodology and ecology are incorporated into economics and harmoniously develop the environment. According to Sinha et al. (2021), ecological economics focuses on environmental and economic challenges that aim to prevent environmental destruction as a result of economic growth. Environmental, economic indicators, environmental development, and environmental energy research are the keys to success. Other methods, such as studying ecological models, are used to understand better how the economy and the environment are intertwined. This helps solve economic ecology issues and uncover the economic ecosystem’s internal significance and requirements. The idea of economic environmentalization is to grow the economy while also protecting the environment on which humans depend, according to Zheng et al. (2021). In order to attain this, environmental protection must be prioritized in all dimensions of environmental protection and economic development actions must be improved. Such improvements include enhancing the production process through advanced technologies, converting harmful toxins liquidated during the production procedure, and utilizing clean energy. To summarize, economics and the environment are mutually supportive of one another. Developing the economy in accordance with the principles of ecology is known as environmental economics. The only way to create a civilization based on ecological principles is to apply environmental economics.

### Green Finance and Environmental Sustainability

Only a small number of research have thus far examined the link between finance and ecology. Environmental sustainability can be attained by arranging funds for solar energy, according to Zhou et al. (2020). Environmental finance/sustainable financing was found to be the most effective method of reducing environmental degradation in a study by Chishti and Sinha (2022). Investing in renewable energy is one way that sustainable finance/green finance promotes new technology and innovation (Ansari et al., 2022). Green bonds (a proxy for green finance) and CO2 emissions have been overlooked in prior studies. Environmentally friendly or pollution-reducing initiatives are the only projects that can be financed with proceeds from green bonds, which are long-term financial securities. Some examples include clean water, solar energy and clean transportation initiatives funded by green bonds.

Green bonds are the best option for green financing technology since they offer long-term capital funding at a low cost. Fossil fuels dominate energy investments. As a result, it is critical to move financial resources away from nonrenewable energy sources and toward sources that reduce carbon emissions (Alola et al., 2022). Investments in green bonds offer a wide range of benefits in addition to their environmental benefits. Introducing green bonds to finance renewable energy projects is particularly attractive. Low-risk, steady-return investments include those in fixed-income securities. Bonds with these characteristics will appeal to domestic and institutional investors, making green financing more attractive. An investor’s risk appetite can be accommodated *via* the issue of bonds, which widens the credit pool (Camana et al., 2021). Direct investing in green technology and clean energy is made possible by spreading liability over a wide range of investors through bonds. Finally, the presence of a secondary market offers investors liquidity and a way out. Those with temporary investment prospects are likewise drawn to this trait. Green bonds are a smart way to increase investments in green technology and renewable energy because of these facts (Camana et al., 2021).

Despite the popularity of green bonds, another option for funding green technology and clean energy projects is equity financing. Investors are unwilling to capitalize on sin stocks that hurt human health and the environment or exploit societal comfort, regardless of the rewards they provide. According to recent years of equities market data, investments in environmental and socially responsible stocks (ESR) have been rising over the last few decades, focusing on the companies’ policies on social, environmental and corporate governance issues, such as human rights. Despite the COVID-19 epidemic, sustainable investments worldwide totaled USD 35.3 trillion, indicating a 15% gain in two years. ESG equities have also been more hardy to market slumps like the global financial crunch, commodities price fluctuations (Saint et al., 2021), or the COVID-19 pandemics (Zheng et al., 2021). Using equity markets to finance green technology and clean energy projects has a number of advantages. It is safe for investors to participate in this market because of the stringent disclosure rules. Dispersion of ownership across shareholders implies that different points of view from various shareholders might be considered while evaluating projects.

## Methodology

### Variable Selection

This study builds a green finance index system that covers five elements, including green securities, green credit, green investment, green insurance, and carbon finance, in order to quantify ASEAN’s green finance more objectively and thoroughly. To advance green innovation and green development, R&D investment is essential. This has been proven to have a threshold effect. Consequently, the threshold variable in this article is the ratio of R&D internal spending to GDP, which represents R&D investment (RDI). Other variables are given in Table 1.

**TABLE 1:** Variable definition.

Variables	Signs	Definition
Green finance	GF	Green finance index system
R&D investment	RDI	R&D internal expenditure/GDP
Green technology	GRT	Clean Technology Index as a proxy for green technology
Human development index	HDI	Urban population/total population
CO2 emission	CO2	CO2 emissions per capita
Foreign direct investment	FDI	Actual Foreign direct investment/GDP
Economic growth	GDP	Total gross domestic product

### Data

Association of Southeast Asian Nations countries are included in the study’s data set, spanning from 2012 to 2019. We used metric tons of CO2 emissions per person, kilograms of oil equivalent per person, and % of total energy derived from combustible, renewable, and waste sources as our clean energy variables. We also looked at the total amount of exports and imports and the money supply to GDP as our indicator for financial development. We used data from World Bank databases for this analysis (WDI).

In terms of data sources, the WDI and the wind databases are used to generate green credit and green security data, respectively. Global Energy Statistical Yearbook provides data on carbon financing and energy input, while Insurance Yearbook provides data on green insurance. The Global Science and Technology Yearbook provides data on R&D spending. Additional information comes from the Global Statistical Yearbook and Global Environmental Statistical Yearbook. For this article’s purposes, we use 2012 as the base year for all price indicators, and we adjust total import and export volumes and real FDI to reflect the current exchange rate in CNY.

### Descriptive Statistics of Variables

The descriptive statistics and pairwise correlations between the various variables are included in Table 2 of the article. It shows that CO2 emissions range from around 1.218 to around 538.12 metric tons, per capita GDP ranges from around 3.17 to around 60.27, and green technology ranges from around 19.56 to around 62.002. Renewable energy consumption ranges from 4.8% to around 3.9% over the sample period.

**TABLE 2:** Descriptive statistical results of variables.

Variable	Mean	Std. Dev	Min	Max
GF	0.297	0.149	0.105	0.826
RDI	1.663	1.138	0.241	6.111
GRT	47.90	8.785	19.56	62.002
HCI	58.19	13.82	30.56	94.08
CO2	30.205	42.23	1.218	538.12
FDI	3.194	5.004	0.0042	32.20
GDP	16.643	10.13	3.17	60.27

Nonrenewable energy consumption has the strongest link with per capita CO2 emissions, whereas financial development has the lowest correlation. However, the foreign direct investment (FDI) is positively connected with CO2 emissions, indicating that increasing renewables can help ASEAN countries reduce their use of nonrenewable energy and hence reduce their CO2 emissions. The analyzed correlation matrix coefficients show that the multicollinearity problem has no significant impact on any estimates.

Table 3 provides descriptive statistics for individual countries. Among ASEAN members, the country of Brunei Darussalam emits the most CO2 per capita, with a 40.322% increase since 2012. Singapore and Malaysia produce significant CO2 emissions in 2020, with per capita emissions at 8.941 and 7.982 metric tons. On the other hand, Singapore saw a 25.317% decrease in CO2 emissions during the same period. Malaysia’s CO2 emissions have risen by 39.545% since 1990. In Thailand, Vietnam, and Indonesia, CO2 emissions have also increased. Cambodia and Vietnam saw the greatest increases in CO2 emissions between 2012 and 2019. The country’s CO2 emissions are still below the average for all ASEAN economies, despite the country’s economic growth.

**TABLE 3:** Description of statistics (Country-specific).

Country	Variables	2012	2019	% Change
Brunei Darussalam	GF	13.253	18.597	40.32%
	GDP	6492.724	8460.589	30.31%
	RDI	53.633	38.784	−27.686**%**
	CO2	108.718	110.197	1.36%
	FDI	36171.81	30717.95	−15.077**%**
Cambodia	GF	0.181	0.566	212.71%
	GDP	276.504	406.173	46.90%
	RDI	5.987	99.986	1570.05%
	CO2	113.743	126.342	11.08%
	FDI	453.969	1374.579	202.79%
Indonesia	GF	1.375	1.956	42.25%
	GDP	742.97	872.424	17.42%
	RDI	18.155	33.154	82.62%
	CO2	69.793	33.19	−52.445**%**
	FDI	2191.574	3756.907	71.43%
Malaysia	GF	5.72	7.982	39.55%
	GDP	2145.964	2941.948	37.09%
	RDI	127.232	134.11	5.41%
	CO2	203.364	116.503	−42.712**%**
	FDI	6890.364	10616.85	54.08%
Philippines	GF	0.891	1.14	27.95%
	GDP	480.604	462.667	−3.732**%**
	RDI	36.265	51.89	43.09%
	CO2	84.9	58.174	−31.479**%**
	FDI	1683.316	3269.671	94.24%
Singapore	GF	11.972	8.941	−25.317**%**
	GDP	5145.886	5007.888	−2.681**%**
	RDI	115.018	132.678	15.35%
	CO2	349.292	320.563	−8.224**%**
	FDI	32597.64	58056.81	78.10%
Thailand	GF	2.906	4.12	41.78%
	GDP	1170.744	1958.152	67.26%
	RDI	93.078	125.033	34.33%
	CO2	120.268	97.929	−18.574**%**
	FDI	3544.442	6199.191	74.90%
Vietnam	GF	0.757	2.002	164.46%
	GDP	379.546	663.076	74.70%
	RDI	39.29	133.923	240.86%
	CO2	111.955	209.323	86.97%
	FDI	804.198	2655.768	230.24%

*Authors’ calculations from the World Development Indicator’s data.*

Brunei Darussalam is ASEAN’s most energy-efficient country. There has been a 30.308% increase in Brunei Darussalam’s kg of oil equivalent per capita consumption since 2012. Energy consumption in Singapore is currently the second-highest in the ASEAN region. Energy consumption in Singapore has decreased between 2012 and 2019, indicating that renewable and cleaner energy sources are better for the economy and the environment. The economies of Malaysia and Thailand are both using a lot of energy to grow. Compared to 2012, Malaysia’s energy consumption has increased by 37.092%. Between 2012 and 2019, Thailand’s energy consumption increased by more than 67%. Among the ASEAN nations, Cambodia uses the least energy. The Philippines’ use of energy decreased by 3.732%.

Cambodia and Vietnam have made the most progress among the ASEAN countries regarding green finance. In 2012, only 5.987% of Cambodia’s GDP was attributed to financial development; by 2019, that number had risen to 99.986%, a gain of 1570.051%. A remarkable increase of more than 240% was seen in the share of financial development in Vietnam’s GDP from 2012 to 2019, rising from 39.290% to 133.923%. Malaysia’s financial development has increased by 5.405% since 2001, which is not encouraging for the country’s prospects for economic growth. Financial development has slowed in Brunei Darussalam by more than 27%, indicating that a weak financial sector has hindered the country’s economic growth and development. Though financial development in Indonesia was improved from 2012 to 2019, the country still holds one of ASEAN’s lowest positions.

According to country-specific data, the ASEAN region’s FDI statistics are mixed at best. FDI fell in all ASEAN economies except for Cambodia, Vietnam, and Brunei Darussalam from 2012 to 2019. There was a 52.445% drop in Indonesia’s FDI index, Malaysia’s (42.712%), and the Philippines’ (31.479%). Thailand and Singapore’s foreign direct investment (FDI) decreased by 8.574% and 8.224% from 2001 to 2020. An 86.770% increase in the FDI index for Vietnam, Cambodia and Brunei Darussalam, respectively. However, according to current data, Singapore is the most open economy in the ASEAN region, while Indonesia is the most closed economy.

Only Brunei Darussalam saw a decrease in environmental sustainability of more than 15% between 2012 and 2019. Singapore’s environmental sustainability is US$ 58,056.810 (in constant terms), while Brunei Darussalam’s is US$ 30,717.950 (in constant terms) (in constant terms). There is also a reasonable level of environmental sustainability in Malaysia and Thailand. Vietnam and Cambodia have both made significant progress in environmental sustainability. ASEAN member economies Vietnam and Cambodia have the lowest environmental sustainability.

The % change in the selected ASEAN economic variables is shown in Figure 1. Changes in Cambodia’s financial progress aren’t shown because of the data’s high observed value.

**FIGURE 1:** % age Changes in the Association of Southeast Asian Nations selected variables between 2012 and 2020.

### Model Specifications

The FMOLS and VECM methodologies are used to determine the impact of green finance on a clean environment and environmental sustainability. Control variables in the model include progress in the foreign direct investment, R&D investment and human development index. Studies such as Ahmad B. et al. (2021), Gao et al. (2021) and others show that financial development and an increase in population (Pop) lead to an increase in CO2 emissions, which is consistent with the findings of previous studies. According to the model’s general specifications:


(1) CO2=F(GF,GDP,RDI,FDI,GRT,HCI)

### Vector Error Correction Modeling

Because of the co-integration of their estimates, it was possible to create a casualty among variables in this study. This, as well as long-term inference, was accomplished through the application of VECM techniques based on Engle and Granger (1987) two-step procedures. Table 2 in the findings section shows the economic performance of the Association of Southeast Asian Nations (ASEAN) in probit and logit terms. The energy efficiency of the countries under consideration in this study is unlikely to be adversely affected by Access or Enimp. It is projected that foreign direct investment (FDI) will play a role in the economic output of ASEAN countries. This is demonstrated by a rise in Chinese investment in the economies of the Association of Southeast Asian Nations. Almost all of China’s and ASEAN’s investments are in energy and transportation, with a little amount in other industries. The total amount of energy produced by ASEAN countries. According to all characteristics, the ASEAN countries with the highest average energy absorption consumption. The VECM technique, which stands for long-term interaction of components, is used to examine how components interact over time. It is possible that the VECM demonstrates short-term causation, but the error correcting word ECT may demonstrate long-term causation eq. (1). Because of this, the VECM equation for economic growth (Y) looks like the following.


(2) $$\begin{array}{c} CO2_{it}=\beta_{0}+\beta_{1}GF_{it}+\beta_{2}RDI_{it}+\beta_{3}HCI_{it}+\beta_{4}FDI_{it}\\ +\beta_{5}GDP_{it}+\in_{it}\\ \mathrm{Where}\text{i}=1,\ldots .,\text{N }\mathrm{and}\text{T}=1,\ldots .,\text{T} \end{array}$$

In order to estimate Eq. (2), we employ an econometric methodology that is divided into three parts. The first step entails determining the degree of integration of each variable that has been employed. Several statistical tests are employed in the econometric literature to determine the degree of integration of a variable. The following are some examples: These are the tests that will be used in this study: Dickey-Fuller Augmenté (ADF); and Phillips-Perron (PP). The next stage will be to investigate the possibility of cointegration relationships between the variables, which may occur over a lengthy period of time once the integration order of the series has been determined for each of the variables. This analysis will be carried out in accordance with the Pedroni test technique. The third stage is concerned with the testing of causality between the variables in the model. The so-called sequential test technique as well as the non-sequential vector error correction model (VECM) procedure will be used in this investigation.

## Results and Discussion

### Unit Root and Co-integration Test

The findings of the ADF and PP unit root tests are presented in Table 4. The findings show no correlation between CO2 emissions, green finance, economic development, FDI, and R&D investment. At this level, these factors are not stable. At 1% and 10%, the degree of significance of clean energy investment and the human capital index is stable. However, when these variables were translated into the first difference, they became stationary at various significance levels. Economic growth and FDI are significant at 10%, CO2 emission at 5%, sustainable environment (SE), clean energy (CE), financial development, and R&D at 1% significance levels, respectively. At both the level and the first difference, clean energy investment and inflation (INF) remain stationary. As a whole, these findings show a mixed bag of happiness, with some factors being I (0), some being I (1), and none being I (). (2).

**TABLE 4:** Unit root test.

		Level				First Difference			
		Intercept		Intercept and Trend		Intercept		Intercept and Trend	
		Statistic	*P*-values	Statistic	*P*-values	Statistic	*P*-values	Statistic	*P*-values
GF	LLC	−1.652	0.115	−0.527	0.242	−5.870	0.000	−4.668	0.000
	IPS	−1.310	0.236	−0.807	0.722	−8.716	0.000	−8.105	0.000
	ADF	40.851	0.113	23.187	0.578	135.617	0.000	119.891	0.000
	PP	78.533	0.275	40.894	0.025	253.255	0.000	655.081	0.000
RDI	LLC	−0.031	0.428	−1.066	0.781	1.250	0.000	−0.787	0.000
	IPS	−5.439	0.880	−3.190	0.880	4.516	0.000	−4.339	0.000
	ADF	11.711	0.877	17.711	0.804	74.568	0.000	67.074	0.000
	PP	7.306	0.880	12.349	0.875	162.105	0.000	155.214	0.000
CO2	LLC	−1.748	0.285	−0.099	0.401	7.031	0.000	−5.953	0.000
	IPS	−1.054	0.778	−1.958	0.869	9.584	0.000	9.407	0.000
	ADF	21.573	0.658	17.877	0.799	148.808	0.000	136.550	0.000
	PP	35.490	0.175	39.283	0.037	287.478	0.000	854.190	0.000
GRT	LLC	−3.702	0.188	−2.105	0.007	−8.260	0.000	−7.631	0.000
	IPS	−0.095	0.402	−0.750	0.173	8.419	0.000	7.429	0.000
	ADF	28.091	0.327	30.695	0.217	128.533	0.000	107.175	0.000
	PP	53.164	0.275	37.908	0.051	195.967	0.000	173.967	0.000
HCI	LLC	−3.155	0.475	4.255	0.000	9.930	0.000	−8.056	0.000
	IPS	−0.163	0.375	3.103	0.000	9.808	0.000	−8.117	0.000
	ADF	30.135	0.239	52.318	0.001	151.870	0.000	117.058	0.000
	PP	29.444	0.267	34.210	0.113	246.523	0.000	210.804	0.000
FDI	LLC	−1.504	0.038	0.115	0.394	−6.533	0.000	−5.537	0.000
	IPS	−0.798	0.720	1.309	0.820	6.714	0.000	5.429	0.000
	ADF	17.788	0.802	16.431	0.833	101.235	0.000	80.760	0.000
	PP	15.374	0.851	10.834	0.878	173.430	0.000	147.233	0.000

Table 5 shows the results of Kao’s residual panel cointegration test (ADF). At the significance threshold of one %, we may reject the original hypothesis that there is no cointegration relationship based on the *p*-Value of 0.0069, which is far less than 0.01. Green finance and clean energy consumption have a significant impact on environmental sustainability. Therefore we can apply a Granger causality test to analyze the link between carbon emissions, economic growth, and green finance.

**TABLE 5:** Co-integration results.

	(1)		(2)		(3)		(4)	
	Coeff.	Significance	Coeff.	Significance	Coeff.	Significance	Coeff	Significance
**Within-dimension**								
V-statistic	5.21	(0.000)*	11.49	(0.000)*	10.65	(0.000)*	32.04	(0.000)*
rho-statistic	–7.74	(0.000)*	10.87	(0.000)*	17.17	(0.000)*	22.31	(0.000)*
PP-statistic	–23.76	(0.000)*	10.65	(0.000)*	14.57	(0.000)*	46.01	(0.000)*
ADF-statistic	17.8	(0.000)*	14.18	(0.000)*	20.69	(0.000)*	25.16	(0.000)*
P-Weighted	14.67	(0.000)*	4.39	(0.000)*	12.03	(0.000)*	19.15	(0.000)*
Rho-Weighted	–9.41	(0.000)*	15.46	(0.000)*	19.4	(0.000)*	19.95	(0.000)*
PP-Weighted	14.9	(0.000)*	17.12	(0.000)*	22.89	(0.000)*	15.79	(0.000)*
ADF-Weighted	10.12	(0.4729)	13.06	(0.000)*	31.15	(0.000)*	8.03	(0.000)*
**Between-dimension**								
Group rho-statistic	2.01	(0.8542)	2.04	(0.7932)	2.00	(0.05819)	2.02	(0.6643)
Group PP-statistic	–2.18	(0.3287)*	–3.47	(0.7932)	–4.94	(0.0000)*	–2.10	(0.2199)*
Group ADF-statistic	–2.29	(0.3496)*	–4.61	(0.6819)*	–4.07	(0.0000)*	–2.18	(0.2018)*

* = p < 0.1.

### Long-Run Estimation

Table 6 shows the long-run estimates of FMOLS and robust least squares for each of the two study models independently. According to the study results, while renewable energy investment has a negative impact on CO2 emissions and ecological footprint, it has a favorable impact on ASEAN’s economic growth. Human capital development index, population, and FDI growth are linked to a reduction in CO2 emissions, a more sustainable natural environment, and increased economic development in the ASEAN region.

**TABLE 6:** Results of long-run estimations.

Variable	GF	RDI	GRT	HCI	FDI	GDP
Brunei	−0.064**	−0.084***	−0.941**	−0.019**	0.263**	0.263***
	(0.358)	(0.000)	(0.008)	(0.021)	(0.019)	(0.002)
Cambodia	−0.088*	−0.067***	−0.425***	−0.048*	0.064**	0.068***
	(0.057)	(0.001)	(0.000)	(0.054)	(0.035)	(0.009)
Indonesia	−0.176**	−0.152***	−0.207**	−0.102**	0.391**	0.391***
	(0.049)	(0.000)	(0.036)	(0.018)	(0.048)	(0.008)
Malaysia	−0.036***	−0.098***	−0.203**	0.072*	0.273**	0.273***
	(0.003)	(0.001)	(0.025)	(0.072)	(0.032)	(0.002)
Philippines	−0.089*	−0.083***	−0.793***	−0.223***	0.454***	0.454***
	(0.079)	(0.002)	(0.002)	(0.002)	(0.000)	(0.000)
Singapore	−0.132***	−0.065***	−2.741***	−0.014***	0.538***	0.538***
	(0.001)	(0.001)	(0.000)	(0.003)	(0.001)	(0.001)
Thailand	−0.024***	−0.277***	−0.183**	−0.107*	0.426***	0.426***
	(0.001)	(0.000)	(0.027)	(0.052)	(0.003)	(0.003)
Vietnam	−0.027**	−0.192***	−1.302***	0.276***	0.124***	0.124***
	(0.014)	(0.000)	(0.000)	(0.001)	(0.002)	(0.005)
Panel	−0.129**	−0.133***	−0.26*	−0.155*	−0.075**	0.778***
	(0.014)	(0.000)	(0.052)	(0.073)	(0.015)	(0.001)

*, **, and *** shows level of significance at 10%, 5%, and 1% level of confidence interval.

Multiple caveats apply to the findings’ interpretation. Starting with a territorial perspective on environmental and resource concerns, the index shows whether nations meet science-based environmental requirements. Environmental norms are shown to be breached, but the index’s indicators cannot reflect the severity of these violations. A good example of this is the outdoor air pollution indicator, which shows how much of the population is exposed to PM2.5 concentrations that are higher than the WHO’s recommended levels. Norm 75 might theoretically be obtained in two countries where one-quarter of the population is subject to pollution levels above environmental standards. At the same time, the other quarter is exposed to pollution concentrations many times greater than the following criteria. As a result, the index’s measures have a territorial rather than a consumption-based perspective. A different perspective might be provided by looking at usage metrics instead.

### Vector Error Correction Modeling Model

These estimators established a long-term, well-balanced link between the two series. According to the VECM model, GDP significantly impacted ASEAN’s CO2 emissions. The strong correlation between GDP growth and CO2 emissions predicts that a 1% increase in GDP will result in a 0.01926% increase in CO2 emissions. The findings of this study are significant, and higher growth rates can result in CO2 emissions. As a result, GDP positively impacts CO2 emissions but was statistically insignificant in the FMOLS estimator (Table 7). According to the VECM estimate, an increase in GDP was accompanied by an increase in the country’s primary production components, including labor, capital, and land. To run these businesses, large volumes of polluting energy must be used, which contributes to the emission of CO2. They support previous studies by Ortega-Arriaga et al. (2021); Sinha et al. (2021), who discovered the link between economic growth and CO2 emissions. We find that GDP is not a significant long-term driver of CO2 emissions, as previously proposed by Khan and Chaudhry (2021).

**TABLE 7:** Casualty test.

	CO2	GF	RDI	GRT	HCI	FDI	GDP	ECT_1
CO2	−	0.138	0.385	0.032	0.199	0.039*	0.159***	0.039
	−	(0.228)	(0.184)	(0.120)	(0.226)	(0.075)	(0.007)	(0.121)
GF	0.080**	−	0.012**	0.060***	0.043*	0.030**	0.036**	0.067***
	(0.012)	−	(0.042)	(0.005)	(0.051)	(0.017)	(0.029)	(0.002)
RDI	0.015**	0.025*	−	0.084***	0.136*	0.059**	0.076**	0.026***
	(0.014)	(0.050)	−	(0.005)	(0.059)	(0.020)	(0.033)	(0.002)
GRT	0.607**	1.258	0.136	−	0.663	0.134	0.548*	0.040***
	(0.013)	(0.587)	(0.472)	−	(0.580)	(0.199)	(0.060)	(0.000)
HCI	0.021**	0.017**	0.133**	0.054	−	0.078**	0.071*	0.055***
	(0.012)	(0.042)	(0.042)	(0.105)	−	(0.017)	(0.076)	(0.002)
FDI	0.039**	0.226	0.139	0.042**	0.230**	−	0.159*	0.024***
	(0.031)	(0.141)	(0.124)	(0.013)	(0.015)	−	(0.053)	(0.001)
GDP	0.047**	0.081	0.198	0.059**	0.126	0.042**	−	0.044**
	(0.013)	(0.139)	(0.113)	(0.043)	(0.112)	(0.037)	−	(0.042)

* = p < 0.1, ** = p < 0.05, *** = p < 0.01.

The study’s findings show that green finance significantly impacts carbon dioxide emissions. An increase in GF will raise emissions by 0.3516% and 0.31094%, respectively, according to estimates from the VECM and FMOLS models. As most ASEAN countries are surrounded by businesses that rely heavily on polluting energy sources, this result is not surprising. Thus, economic activity in ASEAN countries is linked to the large-scale use of unfavorable energy sources, such as coal, natural gas, and the like. This conclusion shows. The country’s emission rate rises as a result of these sources of energy. CO2 emissions in the countries are increased when there is an increase in the processing of goods and services, which is linked to the consumption of large quantities of fossil fuels. According to Tang et al. (2022), environmental sustainability is significantly driven by CO2 emissions, consistent with our findings. On the other hand, opposing our results, Fu et al. (2021) revealed that GF does not influence CO2 emissions, while Sun et al. (2021) discovered an opposite relationship between GF and CO2 emissions, signifying that increasing concept of green finance reduces CO2 emissions.

Both VECM and FMOLS found that FDI had no impact on ASEAN’s CO2 emissions. As shown by the lack of significance of FDI’s impact on CO2 emissions, an increase in FDI in ASEAN countries has little effect on those countries’ emissions. According to this study, people moving to municipalities, which leads to enhanced industrialization, firms’ development, and the formation of roads, hospitals, bridges, and markets, do not affect CO2 emissions. Dong et al. (2021), as well as Salari et al. (2021), all found Inflation (INF) to be a minor source of CO2 emissions. Our findings corroborated theirs. An earlier study by Fu et al. (2021); Khan and Chaudhry (2021), Tang et al. (2022) found that foreign direct investment (FDI) is an important predictor of greenhouse gas emissions.

In the past decade, ASEAN’s green finance has grown significantly, and the overall trend of green finance is positive, according to the ASEAN’s green finance composite index. Overall economic growth increased from 0.2242 to 0.8943, demonstrating that ASEAN’s economy has done well in recent years and has continued to develop. From 0.2077 to 0.8693, the average composite index shows an increasing trend. The robustness economic growth function is larger than the comprehensive index of green finance, demonstrating that an effective development mechanism has been established between the two.

### Discussion

Research on a green premium finds a divided but somewhat positive consensus in the primary ASEAN market. To put it another way, investors are willing to pay more for GF and accept a lower yield in return. Issuers and the growth of the Bitcoin market will benefit from these findings. The GF market may help governments fund zero carbon projects at a lower cost, particularly for bonds that a third party can verify. As more companies learn about the benefits of the green premium, the GF market is expanding. According to this study, non-economic considerations, such as environmental concerns, should be considered when defining bond pricing in the future (Yumei et al., 2021). Green investments, green financing policies, and green financing tools can all benefit from it (such as green bonds). To get the best potential choices for policymakers, further research into this area is timely, pertinent, and of great attention, paying particular attention to the energy sector’s transition and conducting theoretical and empirical debates on the current opportunities and obstacles. These numbers are not insignificant compared to what the Green Climate Fund has raised thus far.

These findings would be altered if different assumptions were made about long-term trends in global GDP, oil prices, and oil supply. However, estimates based on crude oil export taxes give a rough idea of how much revenue could be generated. Mobilizing financial capital for energy efficiency creativities is crucial to combat climate change and meet the rapidly increasing energy requirement. Renewable energy investors face a number of obstacles when it comes to pursuing efficiency and efficiency investments. Therefore green bonds offer a novel way to raise money for both types of projects. The amount of green investment needed to reach this level will increase by 400%. Green bonds may be able to cover this gap in investor assets. A growing number of people are investing in green bonds. The number of countries issuing green bonds is also on the upswing. The Indonesian government has issued around half of the world’s green bonds. It is estimated that green building projects account for more than half of the total invested in green bonds worldwide. In contrast, clean energy production accounts for most of the total invested. In order to attract more investors to green bonds, ASEAN’s offered incentives to bond issuers to cover the costs of third-party audits. Many of ASEAN’s award recipients were first-time issuers drawn to the grant program by regulations that lower the cost of green bond issuing (Zhang et al., 2022).

This analysis concludes that the green credit policy is part of the financial sector’s efforts to promote renewable energy investment. An investigation of the impact of green practices in the form of credit cards and the conditions of credit issuance encourages investment in renewable energy businesses. Eco-friendly renewable energy companies will benefit from this financial aid. It has been shown that green practices in the development of credit cards and credit policies have a significant impact on renewable energy because their major goal is to encourage eco-friendly enterprises. When COVID-19 was in effect, the green securities policy, whether to issue equity or debt securities, significantly influenced investment in renewable energy firms (Xiong and Sun, 2022). Jin et al. (2021) found that investments in renewable energy companies that aim to reduce environmental consequences are encouraged by applying green components in financial securities policies. According to Zhao et al. (2021), the environmental performance of different economic sectors shows that green financial securities have a huge impact on renewable energy project expansion.

The standard of living for humans has been raised thanks to new and creative attempts to improve the environment (Sun et al., 2021). A slow-moving environmental issue, the global financial crisis, can be compared to COVID, a fast-moving and highly stimulated one (Coscieme et al., 2021). In addition to being harmful, this pandemic’s effects on society are worrying. In the post-pandemic era, the gap between supply and demand has widened more than ever before (de Lorena Diniz Chaves et al., 2021). Energy, food, and water scarcity have long been seen as a burden on economies, but the recent rise in health-related concerns has exacerbated this problem. The well-being of society necessitates efforts that are both economical and environmentally beneficial, as well as healthy in terms of protection (Vujanović et al., 2021). In light of the COVID-19 lockout, green financing is being hailed as a possible solution to the global environmental crisis exacerbated by the widespread usage of renewable energy.

COVID-19 has had a profound effect on the economy and industry. Previous years’ corporate and economic problems have been significant, but this virus has utterly destroyed everything. Small businesses are constrained. As a result of the suspension of cross-continental travel and commerce, the economies of all countries have collapsed. COVID-19 is both a medical and financial emergency (Meseguer-Sánchez et al., 2021). Viruses like this one have a devastating effect on businesses. Millions of people worldwide have died as a result of a lack of vaccinations and other preventative medications. All individuals throughout the world have been affected by this pandemic. Employees and employers are increasingly concerned about health-related risks and insurance. Sanitation and the precautionary measures that go along with it have had a profound impact on every industry (Li et al., 2021). Nowadays, workers are more concerned about the cleanliness and health of their workplaces. The only way to combat this global issue is through better planning and the development of less demanding infrastructure on the planet’s resources. Everyone has to break into the business world these days. Creating a green economy is now the only way to run businesses resource-efficient and elegant. Policymakers are developing new and innovative strategies in developed countries to go along with environmentally friendly approaches and COVID-19 preventive treatment options (Tao et al., 2021).

It has also been shown that various insurers’ introduction of green investment strategies has positively impacted green finance investment. According to D’Amato et al. (2021), a study of green finance in developing economies, renewable energy schemes are being monetarily supported by insurers committed to environmental security. The outcomes are also in line with (Shah et al., 2022)’s literary works, which attempt to intricate the role of green investment in finance in enabling the formation of renewable energy companies and enhancing their environmental performance. This study’s outcomes also show that green investment is a strategy for environmentally friendly financial development that continues to promote the use of renewable energy sources even during the COVID-19 period. The goal of green investment is to place funds into environmentally friendly projects. These findings align with previous research by Alataş (2021), which found that providing renewable energy companies with a solid financial foundation improves their performance and encourages economic investment in environmentally friendly projects. A study by Greenfeld et al. (2021) indicated that green economic development contributes significantly to the financial resources of renewable energy firms because of their shared purpose of preserving the environment.

A further study indicated that the corporate social responsibility report published by different corporations, as observed during the pandemic of COVID-19, has a favorable link with investment in renewable energy projects. In agreement with previous research by Zhong et al. (2022), these findings support the hypothesis being advanced. Corporate social responsibility (CSR) reports emphasize the importance of environmental sustainability, so companies invest in renewable energy projects to reduce emissions of hazardous gasses and chemicals by recycling energy resources. These reports are the basis for these studies. A study published by Singh et al. (2021) found that the publication of a business organization’s social responsibility report on a regular basis increases investment in companies that can generate renewable energy and reduce pollution. Finally, the research results show that investments in renewable energy have a favorable impact on economic growth. The findings of Iqbal S. et al. (2021) are consistent with this study. According to this theory, while an economy is developing, all sectors of the economy can invest in initiatives like renewable energy projects that are helpful to their long-term viability.

Innovative business plans necessitate CSR reporting (Can et al., 2021). Every economy relies on the banking sector. Pakistan’s economy is on the verge of collapse, and corruption is the primary culprit (Nabeeh et al., 2021). Corrupt politicians have damaged the Pakistani economy. It is critical that businesses engage in CSR activities (Moussavi et al., 2021). In Pakistan, air pollution is a significant threat. Pakistan is plagued by air, water, and noise pollution (Wiseman et al., 2022). Innovative business planning strategies are required from all policymakers in order to ensure a stable and prosperous economy. It is possible to improve the environment’s health by using environmentally friendly raw materials in factories and waste management programs. Financial difficulties can be overcome with sincere and well-coordinated efforts from people from all walks of life.

## Conclusion and Policy Implications

Green finance, economic growth, energy consumption, and foreign direct investment (FDI) have been studied extensively, but the ASEAN region has received little attention. There is a dearth of a composite metric to describe the entire environmental performance; instead, CO2 emissions are employed as a proxy for environmental quality in earlier studies. This study adds to the growing knowledge on green finance and economic growth, research and development, FDI, green technology innovation, and sustainable development. It also focuses on the ASEAN region. Empirical analyses have also included VECM and FMOLS estimators.

According to research, ecological performance has been shown to improve as a result of green financing. Furthermore, economic expansion has been demonstrated to impact the environment positively. Despite this, ASEAN countries’ environmental performance is deteriorating due to increased energy consumption and foreign direct investment. The study’s findings show that ASEAN financial institutions have lent money to environmentally conscious companies. According to our findings, environmental performance in ASEAN can be improved through the development and implementation of more focused policies and green financing. As a result, the governments of these countries should lend more money to environmentally beneficial and energy-efficient initiatives in the future. Other developing countries around the world should also provide recognition to environmentally and energy-conserving projects. According to the SDGs, this might help accomplish sustainable development and environmental-related goals (SDGs) in 2030. In addition, policymakers should devise policies that sustainably promote economic growth, improving overall environmental performance. Nevertheless, since energy use degrades environmental performance, emerging economies should reduce and regulate their resource usage. To reduce greenhouse gas emissions caused by nonrenewable energy consumption, this study recommends that ASEAN countries in particular and other developing countries, in general, promote renewable energy for the manufacture of goods and home use. Furthermore, the region should support eco-friendly and energy-efficient technology to produce the same amount of goods and services with less energy.

### Practical Implications

Reducing human economic activity’s detrimental externality necessitates global action. Proponents claim that green finance is a critical tool for reducing negative economic consequences while fostering strong economic growth. We advocate the following policies based on the negative association between green finance and CO2 emissions.

1. To encourage the growth of green finance, the ASEAN should implement regulations that use fiscal resources to direct credit funding and social capital into eco-friendly investments, credits, and securities.
2. The government must develop a more efficient and effective green funding system and prioritize green operations in the approval process.
3. Lowered issuance and trading thresholds for eco-friendly securities should be part of government policy in ASEAN undeveloped countries.
4. ASEAN countries should use green financing to raise money to improve the environment.

### Directions for Future Research

In order to attract more investment, our study might be expanded to look at the expansion of green finance into other financial markets from a portfolio viewpoint.

## Data Availability Statement

The raw data supporting the conclusions of this article will be made available by the authors, without undue reservation.

## Author Contributions

Both authors listed have made a substantial, direct, and intellectual contribution to the work, and approved it for publication.

## Conflict of Interest

The authors declare that the research was conducted in the absence of any commercial or financial relationships that could be construed as a potential conflict of interest.

## Publisher’s Note

All claims expressed in this article are solely those of the authors and do not necessarily represent those of their affiliated organizations, or those of the publisher, the editors and the reviewers. Any product that may be evaluated in this article, or claim that may be made by its manufacturer, is not guaranteed or endorsed by the publisher.

## References

[B1] AbbasQ.NurunnabiM.AlfakhriY.KhanW.HussainA.IqbalW. (2020). The role of fixed capital formation, renewable and non-renewable energy in economic growth and carbon emission: a case study of belt and road initiative project. *Environ. Sci. Pollut. Res.* 27 45476–45486. 10.1007/s11356-020-10413-y 32794094

[B2] AbbasiK. R.HussainK.HaddadA. M.SalmanA.OzturkI. (2022). Technological forecasting & social change the role of financial development and technological innovation towards sustainable development in Pakistan : fresh insights from consumption and territory-based emissions. *Technol. Forecast. Soc. Change* 176:121444. 10.1016/j.techfore.2021.121444

[B3] AhmadB.DaL.AsifM. H.IrfanM.AliS.AkbarM. I. U. D. (2021). Understanding the antecedents and consequences of service-sales ambidexterity: a motivation-opportunity-ability (MOA) framework. *Sustainability* 13:9675.

[B4] AhmadM.AhmedZ.YangX.HussainN.SinhaA. (2021). Financial development and environmental degradation: do human capital and institutional quality make a difference? *Gondwana Res.* 105 299–310. 10.1016/j.gr.2021.09.012

[B5] AlataşS. (2021). The role of information and communication technologies for environmental sustainability: evidence from a large panel data analysis. *J. Environ. Manag.* 293:112889. 10.1016/j.jenvman.2021.112889 34087642

[B6] AlolaA. A.AlolaU. V.AkdagS.YildirimH. (2022). The role of economic freedom and clean energy in environmental sustainability: implication for the G-20 economies. *Environ. Sci. Pollut. Res. Int.* 29 36608–36615. 10.1007/s11356-022-18666-5 35066852PMC9079036

[B7] AnS.LiB.SongD.ChenX. (2021). Green credit financing versus trade credit financing in a supply chain with carbon emission limits. *Eur. J. Operat. Res.* 292 125–142. 10.1016/j.ejor.2020.10.025

[B8] Anh TuC.ChienF.HusseinM. A.RamliM. M.PsiM. M. M. S. S.IqbalS. (2021). Estimating role of green financing on energy security, economic and environmental integration of BRI member countries. *Singap. Econ. Rev.* 10.1142/s0217590821500193

[B9] AnsariM. A.HaiderS.KumarP.KumarS.AkramV. (2022). Main determinants for ecological footprint: an econometric perspective from G20 countries. *Energy Ecol. Environ.* 7 250–267. 10.1007/s40974-022-00240-x

[B10] BhardwajA.DagarV.KhanM. O.AggarwalA.AlvaradoR.KumarM. (2022). Smart IoT and machine learning-based framework for water quality assessment and device component monitoring. *Environ. Sci. Pollut. Res.* 1–19.10.1007/s11356-022-19014-335165843

[B11] CamanaD.ManzardoA.TonioloS.GalloF.ScipioniA. (2021). Assessing environmental sustainability of local waste management policies in Italy from a circular economy perspective. An overview of existing tools. *Sustain. Prod. Consumpt.* 27 613–629. 10.1016/j.spc.2021.01.029

[B12] CanM.AhmedZ.MercanM.KaluginaO. A. (2021). The role of trading environment-friendly goods in environmental sustainability: does green openness matter for OECD countries? *J. Environ. Manag.* 295:113038. 10.1016/j.jenvman.2021.113038 34153584

[B13] ChenR.IqbalN.IrfanM.ShahzadF.FareedZ. (2022). Does financial stress wreak havoc on banking, insurance, oil, and gold markets? New empirics from the extended joint connectedness of TVP-VAR model. *Resour. Policy* 77:102718.

[B14] ChienF.ZhangY.SadiqM.HsuC. (2021). *Financing for Energy Efficiency Solutions to Mitigate Opportunity Cost of Coal Consumption : An Empirical Analysis of Chinese Industries.*10.1007/s11356-021-15701-934374014

[B15] ChienF. S.KamranH. W.AlbasharG.IqbalW. (2021). Dynamic planning, conversion, and management strategy of different renewable energy sources: a sustainable solution for severe energy crises in emerging economies. *Int. J. Hydrogen Energy* 46 7745–7758. 10.1016/j.ijhydene.2020.12.004

[B16] ChishtiM. Z.SinhaA. (2022). Do the shocks in technological and financial innovation influence the environmental quality? Evidence from BRICS economies. *Technol. Soc.* 68:101828. 10.1016/j.techsoc.2021.101828

[B17] CosciemeL.MortensenL. F.DonohueI. (2021). Enhance environmental policy coherence to meet the sustainable development goals. *J. Clean. Prod.* 296:126502. 10.1016/j.jclepro.2021.126502

[B18] DagarV.KhanM. K.AlvaradoR.RehmanA.IrfanM.AdekoyaO. B. (2022). Impact of renewable energy consumption, financial development and natural resources on environmental degradation in OECD countries with dynamic panel data. *Environ. Sci. Pollut. Res.* 29 18202–18212. 10.1007/s11356-021-16861-4 34686961

[B19] D’AmatoA.MazzantiM.NicolliF. (2021). Green technologies and environmental policies for sustainable development: testing direct and indirect impacts. *J. Clean. Prod.* 309:127060. 10.1016/j.jclepro.2021.127060

[B20] de Lorena Diniz ChavesG.SimanR. R.RibeiroG. M.ChangN.-B. (2021). Synergizing environmental, social, and economic sustainability factors for refuse derived fuel use in cement industry: a case study in Espirito Santo, Brazil. *J. Environ. Manag.* 288:112401. 10.1016/j.jenvman.2021.112401 33774563

[B21] DongS.XuL.McIverR. (2021). China’s financial sector sustainability and “green finance” disclosures. *Sustain. Account. Manag. Policy J.* 12 353–384. 10.1108/SAMPJ-10-2018-0273

[B22] EngleR. F.GrangerC. W. (1987). Co-integration and error correction: representation, estimation, and testing. *Econometrica* 55, 251–276.

[B23] FangZ.RazzaqA.MohsinM.IrfanM. (2022). Spatial spillovers and threshold effects of internet development and entrepreneurship on green innovation efficiency in China. *Technol. Soc.* 68:101844.

[B24] FengH.LiuZ.WuJ.IqbalW.AhmadW.MarieM. (2022). Nexus between government spending’s and green economic performance: role of green finance and structure effect. *Environ. Technol. Innov.* 27:102461. 10.1016/j.eti.2022.102461

[B25] FengS.ZhangR.LiG. (2022). Environmental decentralization, digital finance and green technology innovation. *Struct. Change Econ. Dyn.* 61 70–83. 10.1016/j.strueco.2022.02.008

[B26] FrancoM. A. J. Q.PawarP.WuX. (2021). Green building policies in cities: a comparative assessment and analysis. *Energy Build.* 231:110561. 10.1016/j.enbuild.2020.110561

[B27] FuF. Y.AlharthiM.BhattiZ.SunL.RasulF.HanifI. (2021). The dynamic role of energy security, energy equity and environmental sustainability in the dilemma of emission reduction and economic growth. *J. Environ. Manag.* 280:111828. 10.1016/j.jenvman.2020.111828 33360740

[B28] GaoM.WangQ.LiL.XiongW.LiuC.LiuZ. (2021). Emergy-based method for evaluating and reducing the environmental impact of stamping systems. *J. Clean. Prod.* 311:127850. 10.1016/j.jclepro.2021.127850

[B29] GreenfeldA.BeckerN.BornmanJ. F.SpatariS.AngelD. L. (2021). Monetizing environmental impact of integrated aquaponic farming compared to separate systems. *Sci. Total Environ.* 792:148459. 10.1016/j.scitotenv.2021.148459 34157536

[B30] HabibaU.XinbangC. (2022). The impact of financial development on CO2 emissions: new evidence from developed and emerging countries. *Environ. Sci. Pollut. Res.* 29 31453–31466. 10.1007/s11356-022-18533-3 35006573

[B31] HuangH.ChauK. Y.IqbalW.FatimaA. (2022). Assessing the role of financing in sustainable business environment. *Environ. Sci. Pollut. Res.* 29 7889–7906. 10.1007/s11356-021-16118-0 34480700

[B32] HuangX.ChauK. Y.TangY. M.IqbalW. (2022). Business ethics and irrationality in SME during COVID-19: does it impact on sustainable business resilience? *Front. Environ. Sci.* 10:275. 10.3389/fenvs.2022.870476

[B33] IqbalS.Taghizadeh-HesaryF.MohsinM.IqbalW. (2021). Assessing the role of the green finance index in environmental pollution reduction. *Estudios de Economia Aplicada* 39:4140. 10.25115/eea.v39i3.4140

[B34] IqbalW.FatimaA.YumeiH.AbbasQ.IramR. (2020). Oil supply risk and affecting parameters associated with oil supplementation and disruption. *J. Clean. Prod.* 255:120187. 10.1016/j.jclepro.2020.120187

[B35] IqbalW.TangY. M.LijunM.ChauK. Y.XuanW.FatimaA. (2021). Energy policy paradox on environmental performance: the moderating role of renewable energy patents. *J. Environ. Manag.* 297:113230. 10.1016/j.jenvman.2021.113230 34303199

[B36] IrfanM.AhmadM. (2021). Relating consumers’ information and willingness to buy electric vehicles: does personality matter? *Transport. Res. Part D Transport Environ.* 100:103049.

[B37] IrfanM.AhmadM. (2022). Modeling consumers’ information acquisition and 5G technology utilization: is personality relevant? *Pers. Individ. Differ.* 188:111450.

[B38] IrfanM.ElavarasanR. M.AhmadM.MohsinM.DagarV.HaoY. (2022a). Prioritizing and overcoming biomass energy barriers: application of AHP and G-TOPSIS approaches. *Technol. Forecast. Soc. Change* 177:121524.

[B39] IrfanM.RazzaqA.SuksatanW.SharifA.ElavarasanR. M.YangC. (2022b). Asymmetric impact of temperature on COVID-19 spread in India: evidence from quantile-on-quantile regression approach. *J. Therm. Biol.* 104:103101. 10.1016/j.jtherbio.2021.103101 35180949PMC8450230

[B40] IrfanM.HaoY.PanjwaniM. K.KhanD.ChandioA. A.LiH. (2020a). Competitive assessment of South Asia’s wind power industry: SWOT analysis and value chain combined model. *Energy Strat. Rev.* 32:100540.

[B41] IrfanM.ZhaoZ. Y.IkramM.GilalN. G.LiH.RehmanA. (2020b). Assessment of India’s energy dynamics: prospects of solar energy. *J. Renew. Sustain. Energy* 12:053701.

[B42] IslamM. M.IrfanM.ShahbazM.VoX. V. (2022). Renewable and non-renewable energy consumption in Bangladesh: the relative influencing profiles of economic factors, urbanization, physical infrastructure and institutional quality. *Renew. Energy* 184 1130–1149.

[B43] JinY.GaoX.WangM. (2021). The financing efficiency of listed energy conservation and environmental protection firms: evidence and implications for green finance in China. *Energy Policy* 153:112254. 10.1016/j.enpol.2021.112254

[B44] JinruL.ChangbiaoZ.AhmadB.IrfanM.NazirR. (2021). How do green financing and green logistics affect the circular economy in the pandemic situation: key mediating role of sustainable production. *Econ. Res. Ekonomska Istrazivanja.* 10.1080/1331677X.2021.2004437

[B45] KhanM.ChaudhryM. N. (2021). Role of and challenges to environmental impact assessment proponents in Pakistan. *Environ. Impact Assess. Rev.* 90:106606. 10.1016/j.eiar.2021.106606

[B46] LiW.YiP.ZhangD. (2021). Investigation of sustainability and key factors of Shenyang city in China using GRA and SRA methods. *Sustain. Cities Soc.* 68:102796. 10.1016/j.scs.2021.102796

[B47] LiZ.KuoT. H.Siao-YunW.The VinhL. (2022). Role of green finance, volatility and risk in promoting the investments in renewable energy resources in the post-covid-19. *Resour. Policy* 76:102563. 10.1016/J.RESOURPOL.2022.102563

[B48] MastiniR.KallisG.HickelJ. (2021). A green new deal without growth? *Ecol. Econ.* 179:106832. 10.1016/j.ecolecon.2020.106832

[B49] Meseguer-SánchezV.Gálvez-SánchezF. J.López-MartínezG.Molina-MorenoV. (2021). Corporate social responsibility and sustainability. A bibliometric analysis of their interrelations. *Sustainability (Switzerland)* 13 1–18. 10.3390/su13041636

[B50] MikhnoI.KovalV.ShvetsG.GarmatiukO.TamošiūnienėR. (2021). Green economy in sustainable development and improvement of resource efficiency. *Central Eur. Bus. Rev.* 10 99–113. 10.18267/j.cebr.252

[B51] MngumiF.ShaorongS.ShairF.WaqasM. (2022). Does green finance mitigate the effects of climate variability: role of renewable energy investment and infrastructure. *Environ. Sci. Pollut. Res.* 1 1–13. 10.1007/s11356-022-19839-y 35386082PMC8986026

[B52] MoussaviS.ThompsonM.LiS.DvorakB. (2021). Assessment of small mechanical wastewater treatment plants: relative life cycle environmental impacts of construction and operations. *J. Environ. Manag.* 292:112802. 10.1016/j.jenvman.2021.112802 34023791

[B53] NabeehN. A.Abdel-BassetM.SolimanG. (2021). A model for evaluating green credit rating and its impact on sustainability performance. *J. Clean. Prod.* 280:124299. 10.1016/j.jclepro.2020.124299 33020685PMC7521472

[B54] NasirM. H.WenJ.NassaniA. A.HaffarM.IgharoA. E.MusibauH. O. (2022). Energy security and energy poverty in emerging economies: a step towards sustainable energy efficiency. *Front. Energy Res.* 10:1–12. 10.3389/fenrg.2022.834614

[B55] NawazM. A.SeshadriU.KumarP.AqdasR.PatwaryA. K.RiazM. (2021). Nexus between green finance and climate change mitigation in N-11 and BRICS countries: empirical estimation through difference in differences (DID) approach. *Environ. Sci. Pollut. Res.* 28 6504–6519. 10.1007/s11356-020-10920-y 32997248PMC7526081

[B56] NingQ. Q.GuoS. L.ChangX. C. (2021). Nexus between green financing, economic risk, political risk and environment: evidence from China. *Econ. Res. Ekonomska Istrazivanja.* 10.1080/1331677X.2021.2012710

[B57] NingY.CherianJ.SialM. S.Álvarez-OteroS.ComiteU.Zia-Ud-DinM. (2022). Green bond as a new determinant of sustainable green financing, energy efficiency investment, and economic growth: a global perspective. *Environ. Sci. Pollut. Res.* 1 1–16. 10.1007/S11356-021-18454-7/TABLES/10PMC873573534993809

[B58] NureenN.LiuD.AhmadB.IrfanM. (2022). Exploring the technical and behavioral dimensions of green supply chain management: a roadmap toward environmental sustainability. *Environ. Sci. Pollut. Res.* 10.1007/s11356-022-20352-5 35460488PMC9034643

[B59] Ortega-ArriagaP.BabacanO.NelsonJ.GambhirA. (2021). Grid versus off-grid electricity access options: a review on the economic and environmental impacts. *Renew. Sustain. Energy Rev.* 143:110864. 10.1016/j.rser.2021.110864

[B60] RaoF.TangY. M.ChauK. Y.IqbalW.AbbasM. (2022). Assessment of energy poverty and key influencing factors in N11 countries. *Sustain. Prod. Consumpt.* 30 1–15. 10.1016/j.spc.2021.11.002

[B61] RehmanA.ZhangD.ChandioA. A.IrfanM. (2020). Does electricity production from different sources in Pakistan have dominant contribution to economic growth? Empirical evidence from long-run and short-run analysis. *Electr. J.* 33:106717.

[B62] SahaT.SinhaA.AbbasS. (2022). Green financing of eco-innovations: is the gender inclusivity taken care of? *Econ. Res. Ekonomska Istrazivanja.* 10.1080/1331677X.2022.2029715

[B63] SaintS.TomiwaA.AdebayoS. (2021). Asymmetric nexus among financial globalization, non - renewable energy, renewable energy use, economic growth, and carbon emissions : impact on environmental sustainability targets in India. *Environ. Sci. Pollut. Res.* 29, 16311–16323. 10.1007/s11356-021-16849-0 34648153

[B64] SalariM.JavidR. J.NoghanibehambariH. (2021). The nexus between CO2 emissions, energy consumption, and economic growth in the U.S. *Econ. Anal. Policy* 69 182–194. 10.1016/j.eap.2020.12.007

[B65] ShahS. A. R.NaqviS. A. A.AnwarS.ShahA. A.NadeemA. M. (2022). Socio-economic impact assessment of environmental degradation in Pakistan: fresh evidence from the Markov switching equilibrium correction model. *Environ. Dev. Sustain.* 10.1007/s10668-021-02013-8

[B66] SinghG.SharmaS.SharmaR.DwivediY. K. (2021). Investigating environmental sustainability in small family-owned businesses: integration of religiosity, ethical judgment, and theory of planned behavior. *Technol. Forecast. Soc. Change* 173:121094. 10.1016/j.techfore.2021.121094

[B67] SinhaA.MishraS.SharifA.YarovayaL. (2021). Does green financing help to improve environmental & social responsibility? Designing SDG framework through advanced quantile modelling. *J. Environ. Manag.* 292:112751. 10.1016/j.jenvman.2021.112751 33991831

[B68] SunY.LiH.ZhangK.KamranH. W. (2021). Dynamic and casual association between green investment, clean energy and environmental sustainability using advance quantile A.R.D.L. framework. *Econ. Res. Ekonomska Istrazivanja.* 10.1080/1331677X.2021.1997627

[B69] SunY.SunH.MaZ.LiM.WangD. (2022). An empirical test of low-carbon and sustainable financing&rsquo;s spatial spillover effect. *Energies* 15:952. 10.3390/EN15030952

[B70] TangC.XueY.WuH.IrfanM.HaoY. (2022). How does telecommunications infrastructure affect eco-efficiency? Evidence from a quasi-natural experiment in China. *Technol. Soc.* 69:101963.

[B71] TangY. M.ChauK. Y.FatimaA.WaqasM. (2022). Industry 4.0 technology and circular economy practices: business management strategies for environmental sustainability. *Environ. Sci. Pollut. Res.* 10.1007/s11356-022-19081-6 35218493

[B72] TaoR.UmarM.NaseerA.RaziU. (2021). The dynamic effect of eco-innovation and environmental taxes on carbon neutrality target in emerging seven (E7) economies. *J. Environ. Manag.* 299:113525. 10.1016/j.jenvman.2021.113525 34438310

[B73] TawiahV.ZakariA.AdedoyinF. F. (2021). Determinants of green growth in developed and developing countries. *Environ. Sci. Pollut. Res.* 28 39227–39242. 10.1007/S11356-021-13429-0/TABLES/11PMC831048733751350

[B74] VujanovićM.WangQ.MohsenM.DuićN.YanJ. (2021). Recent progress in sustainable energy-efficient technologies and environmental impacts on energy systems. *Appl. Energy* 283:116280. 10.1016/j.apenergy.2020.116280

[B75] WangC.LiX. W.WenH. X.NieP. Y. (2021). Order financing for promoting green transition. *J. Clean. Prod.* 283:125415. 10.1016/j.jclepro.2020.125415

[B76] WeiR.AyubB.DagarV. (2022). Environmental benefits from carbon tax in the Chinese carbon market: a roadmap to energy efficiency in the post-COVID-19 era. *Front. Energy Res.* 10:1–11. 10.3389/fenrg.2022.832578

[B77] WeihongJ.KuoT. H.WeiS. Y.Ul IslamM.HossainM. S.TongkachokK. (2021). Relationship between trade enhancement, firm characteristics and CSR: key mediating role of green investment. *Econ. Res. Ekonomska Istrazivanja.* 10.1080/1331677X.2021.2006734

[B78] WisemanN.MoebsS.MwaleM.ZuwarimweJ. (2022). The role of support organisations in promoting organic farming innovations and sustainability. *Malay. J. Sustain. Agric.* 6 44–50.

[B79] WuB.JinC.MonfortA.HuaD. (2021). Generous charity to preserve green image? Exploring linkage between strategic donations and environmental misconduct. *J. Bus. Res.* 131 839–850. 10.1016/j.jbusres.2020.10.040

[B80] XiangH.ChauK. Y.IqbalW.IrfanM.DagarV. (2022a). Determinants of social commerce usage and online impulse purchase: implications for business and digital revolution. *Front. Psychol.* 13:837042. 10.3389/fpsyg.2022.837042 35242088PMC8886314

[B81] XiangH.ChauK. Y.TangY. M.IqbalW. (2022b). *Business Ethics and Irrationality in SMEs?: weivreInweivre.*

[B82] XieM.IrfanM.RazzaqA.DagarV. (2022). Forest and mineral volatility and economic performance: evidence from frequency domain causality approach for global data. *Resour. Policy* 76:102685.

[B83] XiongQ.SunD. (2022). Influence analysis of green finance development impact on carbon emissions: an exploratory study based on fsQCA. *Environ. Sci. Pollut. Res.* 10.1007/S11356-021-18351-Z/TABLES/9PMC878358935066850

[B84] YangC.HaoY.IrfanM. (2021). Energy consumption structural adjustment and carbon neutrality in the post-COVID-19 era. *Struct. Change Econ. Dyn.* 59 442–453. 10.1016/j.strueco.2021.06.017 35317307PMC8506069

[B85] YuJ.TangY. M.ChauK. Y.NazarR.AliS.IqbalW. (2022). Role of solar-based renewable energy in mitigating CO2 emissions: evidence from quantile-on-quantile estimation. *Renew. Energy* 182 216–226. 10.1016/j.renene.2021.10.002

[B86] YumeiH.IqbalW.IrfanM.FatimaA. (2021). The dynamics of public spending on sustainable green economy: role of technological innovation and industrial structure effects. *Environ. Sci. Pollut. Res.* 1 1–19. 10.1007/s11356-021-17407-4 34797541

[B87] ZhangD.AwawdehA. E.HussainM. S.NgoQ. T.HieuV. M. (2021). Assessing the nexus mechanism between energy efficiency and green finance. *Energy Effic.* 14 1–18. 10.1007/S12053-021-09987-4/TABLES/6

[B88] ZhangD.VigneS. A. (2021). The causal effect on firm performance of China’s financing–pollution emission reduction policy: firm-level evidence. *J. Environ. Manag.* 279:111609. 10.1016/j.jenvman.2020.111609 33218832

[B89] ZhangH.GengC.WeiJ. (2022). Coordinated development between green finance and environmental performance in China: the spatial-temporal difference and driving factors. *J. Clean. Prod.* 346:131150. 10.1016/J.JCLEPRO.2022.131150

[B90] ZhaoY.WangC.ZhangL.ChangY.HaoY. (2021). Converting waste cooking oil to biodiesel in China: environmental impacts and economic feasibility. *Renew. Sustain. Energy Rev.* 140:110661. 10.1016/j.rser.2020.110661

[B91] ZhengG. W.SiddikA. B.MasukujjamanM.FatemaN. (2021). Factors affecting the sustainability performance of financial institutions in Bangladesh: the role of green finance. *Sustainability (Switzerland)* 13:10165. 10.3390/su131810165

[B92] ZhongR.RenX.AkbarM. W.ZiaZ.SroufeR. (2022). Striving towards sustainable development: how environmental degradation and energy efficiency interact with health expenditures in SAARC countries. *Environ. Sci. Pollut. Res.* 1 1–18. 10.1007/s11356-022-18819-6 35171428PMC8853387

[B93] ZhouX.TangX.ZhangR. (2020). Impact of green finance on economic development and environmental quality: a study based on provincial panel data from China. *Environ. Sci. Pollut. Res.* 27 19915–19932. 10.1007/s11356-020-08383-2 32232752

